The article "Path Planning and Trajectory Tracking for Automatic Guided Vehicles" was retracted in 2023. Reasons: signs of a paper mill; suspected computer-generated content; unreliable results or conclusions; concerns about the data.

# Path Planning and Trajectory Tracking for Automatic Guided Vehicles

**DOI:** 10.1155/2022/8981778

**Published:** 2022-07-14

**Authors:** Yongwei Tang, Jun Zhou, Huijuan Hao, Fengqi Hao, Haigang Xu

**Affiliations:** ^1^School of Mechanical Engineering, Key Laboratory of High Efficiency and Clean Mechanical Manufacture, Ministry of Education, Shandong University, Jinan 250061, Shandong, China; ^2^Shandong Computer Science Center (National Supercomputer Center in Jinan), Shandong Key Laboratory of Computer Networks, Qilu University of Technology (Shandong Academy of Sciences), Jinan 250014, Shandong, China; ^3^Shandong Shifeng (Group) Company Ltd, Liaocheng 252000, Shandong, China

## Abstract

Automated guided vehicle technology has become a hot area of scientific research due to its increasing use in manufacturing and logistics. Its main features are programming and control, remote computer eye tracking, command receiving and execution, autonomous route planning, and autonomous driving execution of tasks, with the advantages of high intelligence and flexibility. In this work, a simple vehicle model is used to study the route planning and tracking control of automatic guided vehicles. This paper uses wireless communication to find the optimal route planning problem. Using geometric methods, we develop a model of the working environment of the mobile automatic guided vehicle and develop a route finding algorithm. Based on the kinematic model, an advanced routing controller is designed to conduct experimental simulation of two trajectories and verify the effectiveness of the trajectory tracking controller. When the time is after 2 s, the position error is almost completely zero. In the path planning, when the number of iterations is greater than 10, the path length remains constant, verifying the effectiveness of the method in this paper.

## 1. Introduction

The progress of The Times and the rapid improvement of social and economic level make science and technology constantly improve and progress. It has fully entered the daily life and social life of the public and has become an important symbol of a country's strength, and it also plays an irreplaceable role in the development of the market. Among them, the robot technology is the most widely used. It constantly integrates with various industries, affects and interacts with each other, and promotes the innovation, transformation, and upgrading of the industry, which has great value and significance in promoting the sustainable development of the industry. In recent years, with the widening gap in the manufacturing talent market, labor costs are also increasing, and enterprises are in urgent need of a labor force that can replace labor operation and has relatively low production costs. In addition to the in-depth development of robot technology, automatic guided vehicles based on mobile intelligent machine manufacturing technology are being widely used in dry industrial production, logistics and transportation, automobile manufacturing, and many other fields.

The article "Path Planning and Trajectory Tracking for Automatic Guided Vehicles" was retracted in 2023. Reasons: signs of a paper mill; suspected computer-generated content; unreliable results or conclusions; concerns about the data.

Automatic guided vehicles integrate a number of emerging technologies in the existing fields, such as computer control technology, navigation and positioning technology, and communication technology. Compared with the traditional manual work mode, the automatic guided car has a high adaptability and intelligence compared to the external interference. It can be applied in a variety of special working environments, such as radioactive, natural environment dangerous or serious pollution and other workplaces not suitable for manual work, and can better meet the development needs of manufacturing enterprises. However, with the continuous improvement of the market manufacturing level, new problems are also raised for the automatic guided vehicles. The automatic guided vehicles on the market are large, which can only complete the simple transportation work, and the system performance is poor and cannot really improve the automatic production and transportation level of enterprises. In order to fully realize the information and intelligent development of enterprise production and transportation, it is necessary to improve the path planning and track tracking ability of the automatic guided vehicle system.

It explores the functions of path planning and track tracking. It has practical guiding significance and practical significance in promoting the transformation and upgrading of the transportation industry and promoting industrial intelligence and informationization, and provides new ideas for the design and research of automatic guided vehicles. In addition, this research proves that the automatic guided vehicle can complete the tracking under the action of the trajectory tracking controller.

## 2. Related Work

In recent years, many scholars have carried out research on automatic guided vehicles. Leite et al. evaluated the use of an AGV system in an industrial setting and analyzed the pros and cons of the project. He collected data based on actual production systems to develop models and analyze and optimize AGV applications [1]. Yan et al. studied and evaluated the ability of AGV reliability problem. He analyzed the reliability of AGV system through fault tree and evaluated its reliability in vehicle tasks using Petri net method [2]. Setiawan et al. have developed a robot for delivering goods based on an automated guided vehicle. He set the motion of the robot, then controlled it through computer vision, and then used the camera as a sensor to determine the current path in the form of instructions using the navigation system [3]. Weng et al. proposed an improved model with a state classification model and a smooth transition strategy to solve the problems of actuator saturation, parameter selection, and bias relationship of the automated guided vehicle controller [4]. Karimi et al. studied the reliability of machinery in a job shop production system, using automated guided vehicles to handle materials, parts, and other production needs, and a simulation approach to estimate reliability [5]. Gutta et al. reviewed the facility layout design of automated guided vehicles in flexible manufacturing systems, and he addressed many issues related to layout design, location of pickup and delivery points, and process design [6]. To sum up, after several years of exploration, automatic guided vehicles have been deeply studied by many scholars, but the development of the current era has higher requirements for the accuracy and efficiency of automatic guided vehicle path planning and trajectory tracking. Therefore, in order to promote the in-depth development of the application of automatic guided vehicles, the practical research of path planning and trajectory tracking for automatic guided vehicles is urgent.

The article "Path Planning and Trajectory Tracking for Automatic Guided Vehicles" was retracted in 2023. Reasons: signs of a paper mill; suspected computer-generated content; unreliable results or conclusions; concerns about the data.

## 3. Path Planning and Trajectory Tracking of Automatic Guided Vehicles

Automatic guided vehicles are referred to as AGVs, which refer to automated machines equipped with laser equipment or entry equipment [7]. It can design voice paths based on external commands and internal system settings to complete a range of transportation needs. During the transportation process, it mainly uses the battery carried by itself as the kinetic energy. The exterior of the car body is generally provided with protective and auxiliary devices, such as anti-collision devices and assembly spaces.

### 3.1. Working Principle of Automatic Guided Vehicles

The normal operation of the AGV system based on machine technology mainly depends on the CPU processor inside the system. The processor can perform operations such as braking, stationary, real-time monitoring, and safety protection for the AGV, and can even communicate wirelessly with interconnected computers [8]. In the entire transportation process of the automatic guided vehicle, the primary task is to plan and calculate the action path [9]. The path planning of most guided vehicles is assisted by road signs set up on the ground in advance. The guided vehicle recognizes these road signs through the vision system and then enters the system. During the running process, the entered guidance trajectory is tracked to successfully complete the transportation task [10]. It is also applicable in places where the ground environment is more complex, if there are several sub-paths or irrelevant roadblocks on the ground. AGV will activate the safety protection function inside the system and automatically perform actions such as obstacle avoidance and emergency alarm. Then, it tracks the target sub-path according to the identified road signs, and decelerates and accelerates by itself according to the different external environment. In addition to manual remote control operation, AGV driving operation can also realize fully automatic driving. The basic principle is shown in Figure 1.

The article "Path Planning and Trajectory Tracking for Automatic Guided Vehicles" was retracted in 2023. Reasons: signs of a paper mill; suspected computer-generated content; unreliable results or conclusions; concerns about the data.

At present, the automated logistics system consists of automatic production lines, storage rooms, and shelves. This kind of logistics system can not only provide a relatively intelligent action space for automatic guided vehicles, but also monitor the driving status of automatic guided vehicles in real time to escort them. The layout of the modern logistics laboratory is shown in Figure 2.

### 3.2. Overview of Automated Guided Vehicle Systems

This paper mainly introduces the hardware system, vehicle body, electrical device, infrared sensor equipment, and wireless communication device of automatic guided vehicle.

#### 3.2.1. AGV Hardware System

In order to complete the guidance function of automatic guided vehicle, multiple subsystems must cooperate with each other, and many different hardware systems constitute each subsystem. The automatic guided vehicle hardware system is mainly distinguished according to the work and the main functions that each component is responsible for. It is divided into four components, namely, perception layer, decision-making layer, execution layer, and auxiliary layer. The connection of these four-layer hardware modules is shown in Figure 3.

*(1) Perception Layer*. The main task of the perception layer is to collect road condition information, wheel steering information, and planning information in the central controller of the system, and then convert these information data into a set of continuous pulse signals and send them to the driver, in order to realize the braking, running, and control functions of the guided vehicle. It is mainly composed of a camera that collects road condition information, an image acquisition card that stores image data, and a photoelectric encoder.

*(2) Decision-Making Level*. The main task of the decision-making layer is to process and analyze the road condition information, wheel steering information, and planning information in the central controller of the system collected by the perception layer, and then combine the results of the analysis according to the inherent control method inside the system [11]. The decision-making layer is mainly composed of an independent computer and a set of multi-function control boards. The multi-function control boards need to have functions including input and output digital and analog quantities.

*(3) Execution Layer*. The executive layer is the same as the decision-making layer and is mainly connected with the main work content that the upper layer is responsible for. It needs to receive the control instructions issued by the decision-making layer through the driver of the guided vehicle and then control the motor to complete external commands and other tasks within the system. This layer is mainly composed of motors, drivers, deceleration mechanisms, and other equipment.

*(4) Auxiliary Layer*. The auxiliary layer, as the name implies, mainly plays an auxiliary role in the operation of the system in the entire hardware system. For example, it provides light source for the vision system and controls the voltage fluctuation inside the system to ensure the stable operation of the system. The overall equipment of the auxiliary layer consists of a light source and a power source.

The article "Path Planning and Trajectory Tracking for Automatic Guided Vehicles" was retracted in 2023. Reasons: signs of a paper mill; suspected computer-generated content; unreliable results or conclusions; concerns about the data.

#### 3.2.2. AGV Body

Generally speaking, the body structure of an automatic guided vehicle is relatively simple, and its components mainly include functional devices and other auxiliary devices. The functional devices include batteries, operators, etc. Auxiliary devices include lights that provide light, bumpers that protect the body, and six wheels. Steering changes as well as speed control of the AGV are achieved through 6 wheels. Its structure is shown in Figure 4. The wheel in the middle of the body is the driving wheel, which mainly plays a driving role. The front and rear wheels of the body are auxiliary wheels, which are mainly responsible for the load-bearing of the entire body.

#### 3.2.3. AGV Electrical Drive

Its electrical drive device is mainly composed of industrial computer, DC servo motor, motor driver, motion controller, and reducer.

#### 3.2.4. AGV Infrared Sensor Device

The infrared sensor device is set up to prevent the automatic guided vehicle from colliding with irrelevant roadblocks during transportation. Its functions are mainly divided into two categories.

The first type is the anti-collision function; that is, if there is an obstacle in the path when the guided vehicle is carrying out the transportation task, the infrared sensor will immediately receive and transmit the signal, and the CPU controller in the vehicle body system will immediately stop. If the obstacle is removed, the infrared sensor will also receive the signal, and the CPU controller in the vehicle body system will brake the guided vehicle.

The article "Path Planning and Trajectory Tracking for Automatic Guided Vehicles" was retracted in 2023. Reasons: signs of a paper mill; suspected computer-generated content; unreliable results or conclusions; concerns about the data.

The second category is the monitoring function, which can monitor the guided vehicle and determine whether it has reached the target transportation location. When it arrives, the infrared sensor communicates with another sensor that assists in the handling function. After the auxiliary sensor receives the signal of the infrared sensor, the guided vehicle will carry the transported goods.

The basic working principle of the infrared sensor device is based on the reflection principle of infrared light by roadblocks. If the light beam emitted by the sensor is blocked or reflected, there is an obstacle in the path of the guided vehicle. If the infrared light from the sensor is not obstructed in any way, the path is clear.

#### 3.2.5. AGV Wireless Communication Device

The automatic guided vehicle gets in touch with the central console through the wireless communication module during operation [12]. The central console can obtain the location of the automatic guided vehicle in real time through the wireless communication module and perform remote control such as operation mode, and start and stop. The technical indicators of its standard parts are shown in Table 1.

#### 3.2.6. AGV Vision System

The vision system of SRV1 robot has the same principle as that of AGV, which can complete the research on AGV vision. SRV1 is an open-source wireless mobile robot that can transmit live video. Its camera system and image processing system have relatively good performance. SRV1 robot is composed of SRV1 Blackfin camera motherboard, CMOS camera, laser irradiation point, and WLAN802.11 b/g wireless communication module [13].

### 3.3. Automatic Guided Vehicle System Design

#### 3.3.1. Model Predictive Controller Design

Model predictive control is essentially a rolling time domain control strategy. It is different from the traditional control strategy. The traditional control strategy is to continuously apply the state feedback control rate that has been solved offline to the controlled system. The model predictive control is to solve the constrained open-loop control problem in real time in the limited time domain, so as to obtain the optimal sequence [14]. In this paper, the MPC algorithm is used to predict the state of the control system, to solve the numerical solution of the optimization problem, and then to apply the first term of the optimal solution to the control system.

For any sampling moment of the system, no matter what system model is adopted, the measured value will be used as the initial value to predict the future system state. The basic principle is set as the sampling time at the current moment and the measurement value at this time is. Its prediction equation is [15, 16]

(1) $$\begin{array}{c} x\left(k+1\right)=f\left(x\left(k\right),u\left(k\right)\right). \end{array}$$

Among them [17],

(2) $$\begin{array}{c} x\left(0\right)=x_{0},y\left(k\right)=h\left(x\left(k\right),u\left(k\right)\right). \end{array}$$

Among them, *y*(*k*) is the state quantity of the system at the moment, *x*(*k*) is the system control input quantity, and *u*(*k*) is the system output quantity. According to the prediction model, the predicted output value of the system in time domains can be obtained. That is [18],

(3) $$\begin{array}{c} \left\{y_{p}\left(k+1|k\right),y_{p}\left(k+2|k\right),y_{p}\left(k+3|k\right),\ldots ,y_{p}\left(k+p|k\right)\right\}. \end{array}$$

Among them, *y*_*p*_ represents the current time of the system, and the control output of the prediction system at time is predicted, and *y*+*p|k* is the system prediction time domain. In order to reduce the number of independent variables contained in the constrained optimization problem and improve the real time and rapidity of the control algorithm, this paper considers the introduction of the control time domain. If the control time domain is smaller than the prediction time domain, that is, *m* < *p*, and the control variables outside the control time domain satisfy the given control law, the number of independent variables of the system will be determined by the control time domain.

The article "Path Planning and Trajectory Tracking for Automatic Guided Vehicles" was retracted in 2023. Reasons: signs of a paper mill; suspected computer-generated content; unreliable results or conclusions; concerns about the data.

When predicting the control output of the next state of the controlled system, the introduction of control input is considered.

(4) $$\begin{array}{c} \left\{u\left(k|k\right),u\left(k+1|k\right),u\left(k+2|k\right),\ldots ,u\left(k+p-1|k\right)\right\}. \end{array}$$

In trajectory tracking control, the ideal goal is to track the actual output value of the system and eventually converge to the expected output value, that is, the reference trajectory value [19, 20]:

(5) $$\begin{array}{c} \left\{r\left(k+1\right),r\left(k+2\right),r\left(k+3\right),\ldots ,r\left(k+p\right)\right\},\\ J\left(y_{r}\left(k\right),U_{k}\right)=\sum_{i=k+1}^{k+p}{\left(r\left(i\right)-y_{p}\left(i|k\right)\right)}^{2}. \end{array}$$

From this, the basic objective function of trajectory tracking based on MPC algorithm can be obtained. For the automatic guided vehicle, it is necessary to combine the constraints of the guided vehicle itself to improve the objective function and solve it [21].

#### 3.3.2. Automatic Guided Vehicle Trajectory Tracking Controller Design

When the predictive control module of the system tracks and guides the actual path of the AGV, the motion posture of the vehicle body at this moment is set as [22]

(6) $$\begin{array}{c} X={\left[\begin{array}{ccc} X_{0} & Y_{0} & \theta \end{array}\right]}^{T}={\left[\begin{array}{ccc} X & Y & \theta \end{array}\;\right]}^{T}. \end{array}$$

*X* and *Y*, respectively, represent the position coordinates of the center of mass of the car body in the global coordinate system. Taking the linear velocity and angular velocity of the dual steering wheel automatic guided vehicle as the control input, it is represented by the linear velocity and angular velocity of the center of mass of the car body and denoted as [23]

(7) $$\begin{array}{c} u={\left[v_{c\;}\omega_{c}\right]}^{T}={\left[v\;\omega \right]}^{T}. \end{array}$$

If the front and rear wheels of the guided vehicle and the ground in the transportation path belong to a single rolling, it means that the guided vehicle does not slide during transportation. The system kinematics model can be expressed as [24]

(8) $$\begin{array}{c} \left\{\begin{array}{c} \dot{x}=v\;\cos\;\theta ,\\ \dot{y}=v\;\sin\;\theta ,\\ \dot{\theta }=\omega . \end{array}\right) \end{array}$$

Further, the kinematic equation of the automated guided vehicle is shown in [25]

(9) $$\begin{array}{c} \dot{x}=\left[\begin{array}{c} \dot{x}\\ \dot{y}\\ \dot{\theta } \end{array}\right]=f\left(x,u\right)=\left[\begin{array}{cc} \cos\;\theta & 0\\ \sin\;\theta & 0\\ 0 & 1 \end{array}\right]\left[\begin{array}{c} v_{c\;}\\ \omega_{c} \end{array}\right]. \end{array}$$

Since the automated guided vehicle system is a nonlinear and highly coupled system, for such systems, the constrained open-loop control problem can be solved in real time in the limited time domain, which is finally transformed into solving the Hamilton–Jacobi–Bellman equation. Due to environmental constraints or vehicle body maneuverability limitations, it is difficult to obtain accurate analytical solutions by directly solving the equations. Therefore, it is considered to obtain the numerical solution of the constrained optimization problem online, so as to simplify the solution process and make the computing power meet the system requirements of real-time control. Therefore, linear model predictive control is used as an optional solution to solve the AGV trajectory tracking problem.

The article "Path Planning and Trajectory Tracking for Automatic Guided Vehicles" was retracted in 2023. Reasons: signs of a paper mill; suspected computer-generated content; unreliable results or conclusions; concerns about the data.

#### 3.3.3. Establishment of Linear Error Model Based on Quadratic Programming

In order to plan the tracking path of the automatic guided vehicle, a running reference trajectory is established, and any point of the reference trajectory satisfies the state space expression [26, 27]:

(10) $$\begin{array}{c} \dot{x_{r}}=f\left(x_{r},u_{r}\right). \end{array}$$

The reference trajectory state quantity is

(11) $$\begin{array}{c} X_{r}={\left[\begin{array}{ccc} x_{r} & y_{r} & \theta_{r} \end{array}\right]}^{T}. \end{array}$$

The reference input control quantity is

(12) $$\begin{array}{c} u_{r}={\left[v_{r},\omega_{r}\right]}^{T}. \end{array}$$

(*x*_*r*_, *u*_*r*_) is the center of mass coordinates of the reference track vehicle, and [*v*_*r*_, *ω*_*r*_]^*T*^ is the reference heading angle. To linearize the predictive control model, formula (11) is Taylor expanded at the reference trajectory point. Ignoring the higher-order terms and keeping the first-order terms, the linearization error model of the automated guided vehicle can be obtained:

(13) $$\begin{array}{c} \dot{x_{r}}=f\left(x_{r},u_{r}\right)+{\frac{\partial f\left(x,u\right)}{\partial x}}_{|\begin{array}{c} x=x_{r}\\ u=u_{r} \end{array}}\left(x-x_{r}\right)+{\frac{\partial f\left(x,u\right)}{\partial x}}_{|\begin{array}{c} x=x_{r}\\ u=u_{r} \end{array}}\left(u-u_{r}\right). \end{array}$$

That is,

(14) $$\begin{array}{c} \dot{x_{r}}=f\left(x_{r},u_{r}\right)+f_{x,r}\left(x-x_{r}\right)+f_{u,r}\left(u-u_{r}\right). \end{array}$$

Combined with the state space expression, we can get

(15) $$\begin{array}{c} \dot{\bar{x}}=f_{x,r}x^{\prime }+f_{u,r}u^{\prime }. \end{array}$$

Difference between equations (14) and (13) is

(16) $$\begin{array}{c} \dot{x^{\prime }}=\left[\begin{array}{c} \dot{x}-\dot{x_{r}}\\ \dot{y}-\dot{y_{r}}\\ \dot{\theta }-\dot{\theta_{r}} \end{array}\right]=\left[\begin{array}{ccc} 0 & 0 & -v_{r}\sin\;\theta_{r}\\ 0 & 0 & v_{r}\cos\;\theta_{r}\\ 0 & 0 & 0 \end{array}\right]\left[\begin{array}{c} x-x_{r}\\ y-y_{r}\\ \theta -\theta_{r} \end{array}\right]+\left[\begin{array}{cc} \cos\;\theta_{r} & 0\\ \sin\;\theta_{r} & 0\\ 0 & 1 \end{array}\right]\left[\begin{array}{c} v-v_{r}\\ w-w_{r} \end{array}\right]. \end{array}$$

Among them $\dot{\bar{x}}$, refers to the error between the position information of the automatic guided vehicle during transportation and the position information planned in advance by the system controller. Refers to the error between the information collected by the hardware system and the actual road condition information. The linear error model is connected to the state space to become a continuous model, and then the forward difference is used to approximate to obtain the variable discrete error model of the automated guided vehicle when the motion is linear:

(17) $$\begin{array}{c} \left\{\begin{array}{c} x\left(k+1\right)=A_{d}x\left(k\right)+B_{d}u\left(k\right),\\ y\left(k\right)=C_{d}x\left(k\right). \end{array}\right) \end{array}$$

Among them, the linear time-varying matrices are

(18) $$\begin{array}{c} A_{d}=\left[\begin{array}{ccc} 1 & 0 & -v_{r}\sin\;\theta_{r}T\\ 0 & 1 & v_{r}\cos\;\theta_{r}T\\ 0 & 0 & 1 \end{array}\right],\\ B_{d}=\left[\begin{array}{cc} \cos\;\theta_{r}T & 0\\ \sin\;\theta_{r}T & 0\\ 0 & T \end{array}\right],\\ C_{d}=\left[\begin{array}{ccc} 1 & 0 & 0\\ 0 & 1 & 0\\ 0 & 0 & 1 \end{array}\right]. \end{array}$$

Among them, *A*_*d*_ is the sampling period, and *B*_*d*_ is the sampling time.

The article "Path Planning and Trajectory Tracking for Automatic Guided Vehicles" was retracted in 2023. Reasons: signs of a paper mill; suspected computer-generated content; unreliable results or conclusions; concerns about the data.

The nonlinear incomplete system of the linear error model can achieve certain control. It can transform from the initial state to the final state through the limited collection of information data by the system within a given period of time. If the automated guided vehicle is in a nonmoving state, the nonlinear incomplete system cannot be controlled. But as long as the input value is not 0, the nonlinear incomplete system is still the same as the original, and certain control can be achieved. This also means that the linear MPC method is effective to track the transport path of the guided vehicle and use it as the main reference.

## 4. Path Planning and Trajectory Tracking Experiments

The simple control algorithm has the shortcomings of large overshoot, long adjustment time, low control efficiency, and difficult parameter adjustment, which makes it difficult to design the control system [28]. Fuzzy control has the advantages of not needing to clearly know the mathematical model of the control object, imitating human thinking and reasoning, and absorbing expert experience and relatively stable control. In this paper, the fuzzy incremental control algorithm combining the advantages of fuzzy logic reasoning and incremental control is applied to the path tracking control. The fuzzy incremental controller uses the fuzzy logic with expert experience to realize the online self-tuning of parameters and realize the purpose of path tracking adaptive control. The fuzzy incremental controller diagram in this paper is mainly composed of three parts: fuzzy logic inference part, incremental controller, and accumulation part.  Figure 5 shows the block diagram of the fuzzy incremental controller components [29].

When the control path is tracked, the model parameters may change or cannot be determined, and external disturbances will affect the control performance of the controller, so it is necessary to adjust the parameters of the incremental controller in real time during the control process to make the control stable and accurate. The fuzzy incremental controller can adjust the incremental controller parameters in real time through fuzzy reasoning.  Figure 6 shows the fuzzy controller structure [30, 31].

First, we assume that the AGV moves in a limited two-dimensional space. A finite number of known convex polygonal static obstacles are distributed in the AGV's workspace, and there are nodes in the design space that are used to support the AGV and are identified by labels. Based on the above assumptions, the road design problem described here can be described as finding the shortest collision-free path between the start point (assumed to be a node) and the end point (assumed to be a node) when the environmental information is fully known. As shown in Tables 2–4, the coordinates of each node and all possible connection relationships between them are shown.

The article "Path Planning and Trajectory Tracking for Automatic Guided Vehicles" was retracted in 2023. Reasons: signs of a paper mill; suspected computer-generated content; unreliable results or conclusions; concerns about the data.

Experiments show that by developing some specific genetic operators, decimal encoding outperforms binary encoding on most numerical optimization problems. Starting from the starting point, a node that can be connected to the starting point is randomly selected as the next starting point according to the table above. If the number of nodes as the next starting point is large, the probability of these nodes being selected as the next starting point is high and so on until the end point is found.

In order to verify the effectiveness of the algorithm, we have carried out a large number of simulation experiments, and the results are satisfactory. It proposes optimal paths and path length convergence curves as shown in Figure 7. These paths are designed in an obstacle environment, corresponding to different starting and ending points. Experiments show that no matter how complex the environment is, as long as there is a target path, the algorithm can quickly design an optimal path.

In order to verify the feasibility and effectiveness of the above trajectory tracking controller, the trajectory tracking simulation experiment of the automatic guided vehicle is carried out in the MATLAB environment. The simulation results are shown in Figures 8to10.

It can be clearly seen from the experimental results that for straight and circular trajectories, the automatic guided vehicle can complete the tracking under the action of the trajectory tracking controller. The tracking effect is good, the tracking position error is bounded, and it converges to zero within 4 seconds. The simulation results show that the control method is feasible and effective.

## 5. Discussion

Motion planning refers to, given the initial state and the target state, planning a set of movements to enable the automatic guided vehicle to reach the target state without collision. The target state of the automatic guided vehicle can be a fixed point or a movement state. For example, in order to reach the target, the automatic guided car can reach the specified target, and the automatic guided car can adjust the angle error while driving in the process to reach the target point. Then from the curve can also first reverse the angle to the target point, and then directly to reach the target, if there is an obstacle between the current position and the target point, to avoid the obstacle in the process of progress and then reach the target.

The article "Path Planning and Trajectory Tracking for Automatic Guided Vehicles" was retracted in 2023. Reasons: signs of a paper mill; suspected computer-generated content; unreliable results or conclusions; concerns about the data.

The current automatic route planning methods of automatic guided vehicles can be divided into two categories, namely, global route planning and local route planning. In the global planning approach, the most important is the free space method, which is the fundamental stem conformal space. The main local path planning methods are the shortest tangent method, grid method, artificial potential field method, and fuzzy logic algorithm. In traditional methods, the artificial potential field method is the state-of-the-art and most effective programming method. The method is simple and widely used in automatic guided vehicle path planning. In a dynamic changing environment, if global path planning is adopted, this requires more precise global models, and global planning increases the complexity of control. Automatic guided vehicle, always in a dynamic uncertain environment, the feasible path at some point may become infeasible in a very short time, so the significance of global planning is not big. Local path planning not only is simple and ensures the speed of the system, but also improves the decision-making ability of automatic guided vehicles.

In general, a good path planning algorithm should have the following characteristics: 1. rationality: all returned paths are reasonable, or all paths are possible and are accessible by automatically guided vehicles. 2. Completeness: If there is an objective collision-free path from the beginning to the destination, the algorithm can find the motion. A scheduling error is reported if there is no direct-through path nearby. Real-time scheduling algorithm has complex time and storage requirements to meet the movement needs of automatic guided vehicles. There are geometric and physical constraints with multiple restrictions on the movement of automatic vehicles. Geometric constraints are related to the shape constraints of the automatic vehicle, and physical constraints are related to the speed of the automatic vehicle and acceleration. The driving performance requirements of driving multi-purpose automatic guided vehicles have several goals, such as the shortest path, optimal time, optimal safety, and minimum energy consumption. However, there is often a conflict between the two. The optimization algorithm plans the optimal or near-optimal path according to some indicators, such as time, distance, and energy consumption.

The article "Path Planning and Trajectory Tracking for Automatic Guided Vehicles" was retracted in 2023. Reasons: signs of a paper mill; suspected computer-generated content; unreliable results or conclusions; concerns about the data.

## 6. Conclusion

An automated guided vehicle is an unmanned autonomous mobile tool that generates power under its own power and moves under the guidance of equipment. It not only has prominent features in flexible manufacturing systems and automated factories, but also has a wide range of applications in industries such as machinery, automobiles, food processing, and electronics. Countries around the world have incorporated the research on automatic guided vehicles into many advanced technologies, and governments and research institutions of various countries have attached great importance to the development of automatic guided vehicles. In this paper, we propose a simple adaptive controller with fuzzy neural network for tracking control, and the adaptive controller only needs one neural network. To verify the feasibility and effectiveness of the controller, we conduct tracking experiments with two different trajectories. Although fuzzy control is a relatively robust control method, the controller is a fuzzy controller of a single neural network, and its stability needs to be strictly proved in future research work.

## Figures and Tables

**Figure 1:** Working principle of automated guided vehicles.

**Figure 2:** Floor plan of modern logistics laboratory.

**Figure 3:** Automatic guided vehicle system hardware structure.

**Figure 4:** Six-wheeled automatic guided vehicle.

**Figure 5:** Fuzzy incremental controller component block diagram.

**Figure 6:** Fuzzy controller structure.

**Figure 7:** Optimal path and path length convergence curves.

**Figure 8:** Linear tracking situation and attitude error variation curve.

**Figure 9:** Torque change curve and circular tracking situation.

**Figure 10:** Posture error variation curve and torque variation curve.

**Table 1:** Various technical indicators of standard automatic guided vehicles.

Sequence	Technical classification	Parameter index

1	Body size	1200 mm × 550 mm × 800 mm
2	Dead weight	240 kg
3	Maximum load	220 kg
4	Speed	The maximum speed is 0.65 m/s
5	Way of walking	Two-wheel differential
6	Minimum turning radius	480 mm
7	Battery	Lead battery (12 V 38 AH) × 2
8	Communication method	Wi-Fi communication

**Table 2:** 1–4 coordinates and all possible connections between them.

Nodal punctuation	*X*-axis coordinates (m)	*Y*-axis coordinates (m)	Connectable node labels

1	1	5	2, 4, 6
2	1	10	1.5
3	2	1	6.8
4	3	9	2, 7, 9

**Table 3:** 5–8 coordinates and all possible connections between them.

Nodal punctuation	*X*-axis coordinates (m)	*Y*-axis coordinates (m)	Connectable node labels

5	4	12	2, 7, 13
6	6	7	1.3.9
7	7	10	5, 12
8	8	3	3, 6, 12

The article "Path Planning and Trajectory Tracking for Automatic Guided Vehicles" was retracted in 2023. Reasons: signs of a paper mill; suspected computer-generated content; unreliable results or conclusions; concerns about the data.

**Table 4:** 9–12 coordinates and all possible connections between them.

Nodal punctuation	*X*-axis coordinates (m)	*Y*-axis coordinates (m)	Connectable node labels

9	9	7	4, 6, 12, 16
10	9	12	5, 12, 15
11	12,	2	8, 14
12	11	8	7, 10, 16

## Data Availability

This article does not cover data research. No data were used to support this study.
